The article "Motor Imagery and Mental Practice in the Subacute and Chronic Phases in Upper Limb Rehabilitation after Stroke: A Systematic Review" was published in 2023. Journal: Occup Ther Int.

# Motor Imagery and Mental Practice in the Subacute and Chronic Phases in Upper Limb Rehabilitation after Stroke: A Systematic Review

**DOI:** 10.1155/2023/3752889

**Published:** 2023-01-24

**Authors:** Enrique Villa-Berges, Ana Alejandra Laborda Soriano, Orosia Lucha-López, José Miguel Tricas-Moreno, Mar Hernández-Secorún, Miguel Gómez-Martínez, César Hidalgo-García

**Affiliations:** ^1^Physiotherapy Research Unit, University of Zaragoza, Spain; ^2^University of Zaragoza, Spain; ^3^Department of Occupational Therapy, La Salle Higher Center for University Studies, Universidad Autónoma de Madrid, 28023 Madrid, Spain; ^4^Occupational Thinks, La Salle Higher Center for University Studies, Instituto de Rehabilitación Funcional, Madrid, Spain

## Abstract

**Introduction:**

Motor imagery and mental practice can be defined as a continuous mechanism in which the subject tries to emulate a movement using cognitive processes, without actually performing the motor action. The objective of this review was to analyse and check the efficacy of motor imagery and/or mental practice as a method of rehabilitating motor function in patients that have suffered a stroke, in both subacute and chronic phases. *Material and Methods*. We performed a bibliographic search from 2009 to 2021 in the following databases, Medline (PubMed), Scopus, WOS, Cochrane, and OTSeeker. The search focused on randomized clinical trials in which the main subject was rehabilitating motor function of the upper limb in individuals that had suffered a stroke in subacute or chronic phases.

**Results:**

We analysed a total of 11 randomized clinical trials, with moderate and high methodological quality according to the PEDro scale. Most of the studies on subacute and chronic stages obtained statistically significant short-term results, between pre- and postintervention, in recovering function of the upper limb.

**Conclusions:**

Motor imagery and/or mental practice, combined with conventional therapy and/or with other techniques, can be effective in the short term in recovering upper limb motor function in patients that have suffered a stroke. More studies are needed to analyse the efficacy of this intervention during medium- and long-term follow-up.

## 1. Introduction

The World Health Organization (WHO) defines stroke as the clinical syndrome characterised by the rapid development of symptoms and/or local or generalised signs of neurological affectation, which lasts more than 24 hours and can even lead to death, without other apparent cause than a vascular origin [1].

A stroke causes neurological deficits in various domains of brain areas: motor, sensory/perceptive, visual, language, cognitive, intelligence, and emotion. In the motor area, the most frequent syndrome is hemiplegia or hemiparesis [2, 3]. Motor deficits occur predominantly unilaterally, contralateral to the injured side. Different areas of the brain can assume their functions through a spontaneous biological recovery and then move on to a phase of compensation. The phases of stroke have a process of change, and biomarkers will help to improve future treatments and will have to identify the effect on these phases [4].

The article "Motor Imagery and Mental Practice in the Subacute and Chronic Phases in Upper Limb Rehabilitation after Stroke: A Systematic Review" was published in 2023. Journal: Occup Ther Int.

Within this review, we can define the periods of analysis of the studies in 2 phases: the late subacute phase, which includes from 3 months to 6 months, and the chronic phase, which encompasses more than 6 months of evolution of the disease [4].

Between 30% and 66% of the individuals that have a stroke do not reach satisfactory motor recovery of the affected upper limbs following rehabilitation; this is one of the main causes of disability and produces great limitations in the activities of daily living (ADLs) [5, 6].

There are many definitions from authors that define motor imagery (MI) and mental practice (MP) as a continuous mechanism in which the subject tries to emulate a movement using cognitive processes, without actually performing the motor action [7–9]. In other words, MI consists of the mental representation of the movement, without the actual presence of it. It is a complex cognitive operation that is possible thanks to the use of sensory and perceptive processes that allow an individual to reactivate specific motor actions in the working memory [10]. In the case of MI, reactivation happens when the movement is imagined rather than performed, implying a voluntary impulse. We can generate a movement in this way without needing to perform it, intending to acquire and optimise motor skills [10]. This theory proposes that MI, the observation of the movement and the performance of the movement, share a central nervous function that corresponds among them [11].

These techniques are based on the theory of mirror neurons and demonstrate that people can produce plastic changes in the functionality of hand movements. Several studies have identified patterns in brain activation that occur during MI and found that MI largely activates regions including the frontoparietal network, subcortical and cerebellar regions, anterior intraparietal cortex, primary motor cortex (M1), bilateral supplementary area (SMA), and premotor area (PMA) [12]. Another study [13] showed that the use of MI improves a patient's upper limb motor functions and activation areas mentioned in the previous study.

People can also develop MP using images of limb movements, which can make it easier for people that have suffered a stroke to recover motor function. Commitment and motivation are essential for participating in the MI training program [14].

The article "Motor Imagery and Mental Practice in the Subacute and Chronic Phases in Upper Limb Rehabilitation after Stroke: A Systematic Review" was published in 2023. Journal: Occup Ther Int.

The theory of sports science was the origin of MP. This theory establishes that rehearsing can improve the acquisition of motor skills [15]. MP is a method of training during which a person cognitively rehearses a physical skill using motor images, without the presence of physical movements, in order to improve the performance of motor skills [16], when an individual can access the perceptive information from the memory, MP [17].

Both MP and MI can provide an effective strategy to facilitate motor recovery in patients with brain lesions. This is especially true during the first stage of rehabilitation, when full participation in occupational and physical therapy programs may not be possible due to excessive motor weakness of the upper limbs [18]. Studies such as [19] show results indicating a preserved interhemispheric balance of patients in the subacute stage by activating cortical motor areas during MI.

Likewise, the scientific literature indicates that both MP and MI can be effective interventions in chronic phases, because there can also be limitations in the functional mobility of the upper limbs. MI might contribute to motor recovery in chronic stroke patients through the following network reorganization, i.e., promoting the efficiency of regional neuronal communication, and the reorganization of intrinsic functional connectivity of the ipsilesional M1, involving a widely distributed motor network in both hemispheres (H. [20]).

The objective of this systematic review was to analyse and check the efficacy of motor imagery and/or mental practice as a method of rehabilitating motor function in patients that have suffered a stroke, in both subacute and chronic phases.

## 2. Material and Methods

### 2.1. Design

We searched bibliographic databases through November 2021. The search consisted of finding randomized clinical trials in which the main subject was rehabilitating the motor function of the upper limb in people that had suffered a stroke, using the MI and/or MP techniques alone or combined with other therapies. Systematic reviews of reviews were conducted, as well as a synthesis of the findings of all systematic evidence published based on Smith et al. [21]. This systematic review was carried out following the recommendations of the Preferred Reporting Items for Systematic Reviews and Meta-Analyses (PRISMA) guidelines [22], with registration number CRD42021160215 in the prospective register of systematic reviews (PROSPERO).

### 2.2. Search Strategy

#### 2.2.1. Search Limits

For the article search, we applied the following filters for study inclusion: randomized clinical trials (RCTs) and controlled clinical trials, studies in humans, people with ages more than 18 years, articles published in the last 12 years, and manuscripts written in English or Spanish.

The article "Motor Imagery and Mental Practice in the Subacute and Chronic Phases in Upper Limb Rehabilitation after Stroke: A Systematic Review" was published in 2023. Journal: Occup Ther Int.

Two authors performed the bibliographic search and evaluated the titles, abstracts, and complete texts, following the eligibility criteria. If there were any disagreements or doubts, these 2 authors consulted a third author to resolve the discrepancies.

We searched for articles in the main bibliographic databases: PubMed, Web of Science (WOS), Cochrane, Scopus, and OTSeeker. The search terms or keywords used to gather the data and select the information were the following: “stroke”, “motor imagery”, “mental practice”, and “upper limb function”.

#### 2.2.2. Inclusion and Exclusion Criteria

The articles selected included patients diagnosed with stroke and with the upper limb affected, having MI or MP as the only treatment modality or together with other interventions, in both subacute and chronic phases. The late subacute phase includes from 3 months to 6 months, and the chronic phase encompasses more than 6 months of evolution of the disease, once the motor deficits start to settle into a definite pattern.

We excluded articles that referred to pathologies other than stroke or in which the main intervention objective was not to improve upper limb functionality. We also excluded articles on treatment interventions with children. Lastly, we ruled out articles that did not fulfil a methodological quality criterion, based on the Physiotherapy Evidence Database (PEDro) scale. Only the final results of articles with moderate and high methodological quality according to the PEDro scale criteria were obtained during the bibliographic search.

#### 2.2.3. Data Extraction Process

First, the two independent reviewers performed data analysis, assessing the relevance of the reviews regarding the study questions and objectives. This initial analysis was performed based on information from each study's title, abstract, and keywords.

We gathered the following information for each study: (1) author and year of publication, (2) study objectives, (3) sample characteristics, (4) group protocols, (5) measurement variables, and (6) results. After that, all the information was analysed and then summarised (Table 1).

### 2.3. Assessment of Methodological Quality

The methodological quality of the randomized clinical trials was assessed using the PEDro scale. It is one of the clinical trial assessment tools utilised the most in studies that focus on stroke rehabilitation [33].

It is considered a very reliable scale and is also recommendable for the systematic review of controlled clinical trials. It defines, with a low risk of bias, articles that obtain a score above 6 points as high quality, those that achieve between 4 and 6 points as moderate quality, and articles with scores of 3 points or less as low quality [34].

The article "Motor Imagery and Mental Practice in the Subacute and Chronic Phases in Upper Limb Rehabilitation after Stroke: A Systematic Review" was published in 2023. Journal: Occup Ther Int.

In our review, we will analyse the articles that obtain a score equal to or higher than 6 points, which are considered high-quality articles, with the exception of the article of [31], which is a nonrandomized study and therefore penalizes its methodological quality, but the authors believe that it should be included, since we could lose relevant information.

## 3. Results and Discussion

### 3.1. Internal Validity of the Articles

In this systematic review, we assessed 11 studies. The flow diagram is shown in Figure 1.

These consisted of 9 randomized clinical trials (RCTs), 1 randomized cross-over trial [25], and 1 nonrandomized clinical study [31]. All the studies complied with the criteria for inclusion and exclusion. These 6 articles obtained a high methodological score in the reference list [23, 24, 26, 27, 30, 32] while these 4 articles obtained a moderate methodological quality based on the PEDro scale (Table 2) [25, 28, 29, 35]. Only one study [31] cannot be analysed due to the type of study.

In the specific case of the study [30], since it is a quasiexperimental design, in which we do not have a control group as such, it is difficult to define the efficacy of MI/MP. Instead, it gives us another point of view on how to administer MI/MP and that a distributed practice could be beneficial, compared to a mass practice, for the improvement of upper limb function.

### 3.2. Description of the Study Samples

The sample size of the studies ranged from 10-19 patients [26, 28, 29] to 20-38 patients [24, 25, 31, 32, 35]. There were only 3 studies with more than 40 patients [23, 24, 30]. As for stroke evolution, in this review, we divided the studies into 2 groups: articles applying the rehabilitation interventions during the subacute phase of the lesion [24–27, 30, 32, 35] and the remaining ones applying interventions during the chronic phase [23, 28, 29, 31]. In all the studies, the sample consisted of adult patients, distributed evenly between men and women, which presented an affectation of the upper limb due to hemiparesis or hemiplegia.

In terms of lesional side involvement, there is heterogeneity in how the sample is described. There are 2 studies that mention that all their subjects are right-handed, as assessed by the Edinburgh scale [26, 35]. Another study does not mention the involvement of the injured side in the upper extremity in its sample [25]. One of the studies refers to the affected cerebral hemisphere, which has an impact on the limitation of movement of the damaged upper limb [24]. Finally, the rest of the studies describe the affected side of the upper limb, whether it is the right or left lesional side, where there is hardly any predominance of one side over the other [23, 27–32].

The article "Motor Imagery and Mental Practice in the Subacute and Chronic Phases in Upper Limb Rehabilitation after Stroke: A Systematic Review" was published in 2023. Journal: Occup Ther Int.

Due to the variability in describing the involvement of the injured or dominant side of the participants in each study, it is difficult to obtain an approximate conclusion of the possible recovery of the upper limb.

### 3.3. Description of the Study Interventions

In all the studies, the intervention method carried out for the MI and/or MP technique was specified. A therapist supervised the patients, guiding them and ensuring that the instructions were followed. The process commenced with a period of relaxation and becoming aware of the limb affected. The patients kept their eyes closed or covered, focusing on the limbs in a first-person view; that is, the patients visualised the hand and arm as if they were seeing their own body parts with their own eyes. After acknowledging the mental image of the upper limb affected, the patients began imaging that they were making a few simple movements, such as flexion of just their shoulder or their elbow or both, flexion and extension of the wrist, opening and closing the hand, separating the fingers, and pressing the tips of 2 fingers together. The patients then continued imagining more dynamic movements aimed at specific ADLs, such as picking up a bottle of water and drinking and putting on a t-shirt.

All the studies included in this review also featured conventional physiotherapy and/or occupational therapy treatment. In the articles, this treatment was described as stretching exercises or neurodevelopment techniques and techniques for progressing towards maximum independence in ADLs.

In 7 of the studies performed in the subacute phase, the researchers compared an experimental group (EG) that did MI or MP combined with conventional treatment (physiotherapy and occupational therapy) and a control group (CG) that performed only the conventional treatment [24–27, 30, 32, 35].

In 4 studies on patients in the chronic phase, the investigators also compared an EG consisting of patients that did MI and/or MP combined with conventional treatments, with a CG that performed only conventional treatment [28, 29, 31]. In their study, [30] distinguished between distributed and massive MP in different groups, and they introduced an audio recording in the MP process. The distributed MP consisted of carrying out 20 minutes of MP 3 times a day; in contrast, the massive MP was performed in a single 60 min session every day.

The article "Motor Imagery and Mental Practice in the Subacute and Chronic Phases in Upper Limb Rehabilitation after Stroke: A Systematic Review" was published in 2023. Journal: Occup Ther Int.

In general, there was no consensus on treatment duration and frequency. Treatment lasted for periods ranging from the 3 weeks [24] used to the 6 weeks [23] proposed. A treatment of 4 weeks was used the most among the studies analysed, with either a more intensive frequency of sessions 5 days a week or alternating 3 days a week.

In all the studies, the patients were assessed before the intervention and posttreatment. Not all the articles included a later follow-up; in those that did, it varied between 1 month, 3 months, and 12 months [23].

### 3.4. Description of the Results of the Studies

One of the most widely used assessment instruments is the Fugl-Meyer upper extremity (FMA-UE), which appears in 9 of the 11 studies.

Following the ICF criteria, to assess body functions, FMA-UE, as well as the goniometer or Modified Ashworth Scale (MAS), may be used.

To analyse activity, the most commonly used were the Wolf Motor Function Test (WMFT), Action Research Arm Test (ARAT), Box and Blocks Test (BBT), Jebsen Taylor Hand Function (JTTHF) test, Motricity Index (MI), and Modified Barthel Index (MBI), among others.

In terms of participation, these studies used the Stroke Impact Scale (SIS), Motor Activity Log-30 (MAL-30), and Canadian Occupational Performance Measure (COPM), among others.

The next sections detail the most relevant results of the studies.

#### 3.4.1. Articles to Be Analysed

In the articles focusing on the subacute phase without combining techniques in the EG, statistically significant differences were found between groups. The most representative study variables were the FMA-UE and ARAT [27, 32, 35]. It is notable that in their study, [23] found that the patients maintained the positive results in the Frenchay Arm test over time, up to 12 months of follow-up. In the rest of these subacute studies, no statistically significant results or differences were obtained between groups [25–27, 30].

The articles on studies carried out in the chronic phase without combining techniques in the EG showed statistically significant changes in the measurements from the FMA-UE [28, 29, 31, 36], as well as in other variables from instruments such as the ARAT, BBT, and COPM.

Most of the 11 studies that included both phases obtained statistically significant positive results in the recovery of upper limb function. However, in the majority of these studies, the researchers did not specify follow-up after the postintervention period, except for [23] in their study. This is an important factor to consider, because it means that we cannot state that the changes produced in upper limb function would be maintained over time. More studies that include follow-up after the intervention are needed to make it possible to analyse the continuance of the benefits of the technique once the treatment has ended.

The article "Motor Imagery and Mental Practice in the Subacute and Chronic Phases in Upper Limb Rehabilitation after Stroke: A Systematic Review" was published in 2023. Journal: Occup Ther Int.

During the first 6 months after a stroke, patients experience a spontaneous recovery [37]. There is greater neuroplasticity in this period of time, which helps to reorganize and create new synapses; mental practice and/or motor imagery during this period could hypothetically promote this neuronal plasticity [38].

It has been shown that, in the chronic phase, neuroplastic changes also continue happening, helping cortical reorganization even though the lesion has lasted for years [38], with statistically significant results in the treatments, as the studies discussed in this review [28–32]. Consequently, this is a phase and a subject that needs further research. This would strengthen the performance of interventions, among which MI and/or MP could be included.

Therefore, we can conclude that MI/MP intervention in both the subacute and chronic phases is an effective technique in improving the functionality of the affected upper limb, and not only in the acute phase, as has been analysed up to now, given the evidence analysed in this review.

### 3.5. Description of the Study Conclusions

Most of the studies agree that MI and/or MP treatment combined with traditional treatment is more effective in upper limb motor recovery (general motor movements, speed and coordination of movement, and, above all, in the integration of these changes in carrying out ADLs) than intervention with only conventional treatment, in both the subacute and chronic phases [23, 24, 28, 31, 32, 35].

The MI/MP technique does not require great economic investments and can be performed anywhere, because no special equipment is needed. It is safe, given that the technique can be repeated many times without great physical effort.

The benefits provided by mental practice (MP) and/or motor imagery (MI) in upper limb rehabilitation after a stroke seem promising. However, there are systematic reviews and meta-analyses that tell us that the technique is not effective on its own [39], although it can be beneficial if combined with conventional therapies or with other types of techniques [16, 40]. Further research is needed about the approach to the appropriate dose of sessions and the effects of the visual and kinaesthetic images, as well as the perspective of the image, during the mental depiction. Researchers in the field need an assessment tool to analyse and quantify the patients' capacity to represent the affected limb using mental practice. Whether the benefits obtained last over time also has to be established, there are barely any studies that include follow-ups, except for the study of Annick et al. [23]. Finally, highlight that none of the included studies analysed the benefits obtained in upper limb motor recovery in occupational tasks.

The article "Motor Imagery and Mental Practice in the Subacute and Chronic Phases in Upper Limb Rehabilitation after Stroke: A Systematic Review" was published in 2023. Journal: Occup Ther Int.

Comparing the information with other systematic reviews, we have detected that in 3 of the studies analysed [5, 41, 42], integration and change between functionality and ADLs were not analysed. However, in 7 studies [23, 24, 27–29, 31, 32], these associations have been related. It should be noted that in the Cochrane review [43], there is a low certainty of evidence indicating that it is possible that ADLs do not improve with MP.

Analysing and comparing the studies that make up this review and other systematic reviews, we can expose that the ability to imagine is not systematically evaluated with an assessment tool in most studies, making it difficult to obtain real data on whether this ability to imagine is happening or is being executed correctly. Therefore, it should be urged that in the next RCTs, the ability to imagine should be continuously assessed by means of validated assessment tools or diagnostic tests, so that they can clarify the efficacy of MI/MP.

### 3.6. Limitations of the Studies

There were biases in selection in the various studies analysed. There were no homogeneity and consensus in the protocols, with a strong, detailed methodology, unified measurement parameters, and a schedule for efficiency. In addition to the differences in study design and methodological quality, the articles analysed varied with respect to sample characteristics, intervention protocols, and result measurements (Tables 1 and 2).

Focusing specifically on intervention protocols, all the studies combined physical practice and mental evocation, although there were differences among them. Examples are in how image evocation was facilitated (audio tapes, spoken instruction, or television images), the type of imagery used (internal or external), the tasks that were practiced, and the length and intensity of the treatment sessions.

The extent to which the samples varied, in both age range and location of the stroke lesion, and even the exclusion of different stroke subgroups, makes it difficult to compare the studies. With respect to the type and location of the lesion, 4 studies mentioned only that it had to be the first stroke diagnosed, without considering the location [24, 29–31]; 2 studies indicated that it had to be the first stroke and with unilateral lesion diagnosed [26, 28]; other study considered only ischemic stroke with unilateral affectation [25]; 1 study considered that both the lesion and the dominant hand had to be the right hand before the stroke [35]; and others did not discriminate as to the type of lesion or location but alluded to lesion location as an excluding factor, such as the article of Page et al. [30], which excluded individuals having affectation of the parietal lobe because such damage is related with difficulties to evoke motor images using MP. In contrast, 1 study considered lesion location in the criteria for inclusion. In their study, Hua Liu et al. [26] included patients with a first stroke diagnosed in the subcortical area.

The article "Motor Imagery and Mental Practice in the Subacute and Chronic Phases in Upper Limb Rehabilitation after Stroke: A Systematic Review" was published in 2023. Journal: Occup Ther Int.

Most of the studies have small samples that cannot be representative of the population, due to the difficulty in finding an appropriate sample and people willing to participate in the study [23–26, 28, 29, 31, 32, 35]. We can find that in 7 of the studies, the calculation of the sample size was not carried out. Variable recruitment of the study sample was present. In the subacute phase, recruitment was performed in hospitals ([24, 25, 27, 35]) and hospital and rehabilitation centers [23] and not reported [26]. In the chronic phase, recruitment was performed in the hospital [32], in the hospital and rehabilitation centers [31], with brochures and support from stroke groups [28], and not reported [29].

There are differences in the recruitment according to the recovery phase of the patient (subacute or chronic), which makes it difficult to extrapolate the results to a certain phase of recovery.

There is also a notable lack of information about the area of lesion most affected and the type of stroke (ischemic and haemorrhagic). These 2 factors might have influenced the results, and we suggest that researchers consider them in future studies, as Azad et al. [31] did. They also mentioned the limited number of treatment sessions per week, the intervention intensity, and the number of repetitions needed, which these authors believed were insufficient to achieve motor learning, based on their observations [26].

Although there are different measures to assess MI, it has been impossible to establish its predictive value [44]. As an intervention based on people's imagination, it is difficult to control and assess in a concrete way the capacity that an individual possesses to develop it [5]. None of the studies analysed assessed the entire sample for the capacity to image visually and kinaesthetically. Consequently, we do not know with certain accuracy the capacities the patients had for representing the affected upper limb in the primary motor and somatosensory cortex.

In the studies, the specific training required in this technique for the therapist was not indicated. In addition, the type of motor imagery, kinaesthetic or internal (first person) or visual or external (third person), was not considered; kinaesthetic motor imagery is more effective [45].

The article "Motor Imagery and Mental Practice in the Subacute and Chronic Phases in Upper Limb Rehabilitation after Stroke: A Systematic Review" was published in 2023. Journal: Occup Ther Int.

All of this represents a problem. Although it has been suggested that many people still preserve their capacity to mentally represent the movements of the affected upper limb after suffering a stroke [46], it seems that certain brain lesions (for example, in the parietal lobe [16]) can cause an inability to evoke motor images [47]. A simple change in the instructions about the images to imagine (first or third person) and in the real posture of the hand (holding an object in the hand and the spatial situation of that object) would have a strong impact on the time and precision of the response from the individuals that have suffered a stroke [48].

We also feel that the cognitive capacities that the participant needs (in both attention and concentration) have to be mentioned [49], and there are some review articles that do not include among their inclusion criteria an assessment tool that evaluates the cognitive capacity of the participants [23, 26, 35]. The reason is that, if the individuals do not possess these capacities, those participants might not be people that could benefit from this treatment.

Lastly, the lack of uniformity in the use of terminology in the databases might represent a limitation, given that there is not a single, unique term corresponding to MI or MP. This diversity of terms, together with the language criterion (English and Spanish), may have caused the loss of studies to include in this systematic review.

## 4. Conclusions

Motor imagery and/or mental practice have obtained promising results in improving upper limb function after a stroke, while also improving movement integration and patient participation in activities of daily living; when these techniques are combined with conventional treatment and/or other techniques, they constitute an appropriate complement. Researchers need a greater number of studies that analyse adequate MI/MP scheduling, patient suitability and homogeneity, the way the imagination is presented, and the durability of the positive results over time.

We can conclude that MI/MP intervention in both the subacute and chronic phases is an effective technique in improving the functionality of the affected upper limb and not only in the acute phase.

## Figures and Tables

**Figure 1:** Result strategy flowchart.

**Table 1:** Summary of the characteristics of the studies analysed.

Study	Aim	Sample characteristics	Procedure	Outcome variables	Results
[24]	Design: CT not randomized To investigate the effect of MI training with sensory feedback on sensory-motor function of the upper extremity in patients with chronic stroke	Stage: chronic *n*: 30 *n* (IG): 15 *n* (CG): 15	12ss × 3 v/wk × 4 wk IG: 45-60 min IM + conventional rehabilitation CG: conventional rehabilitation Assessment: baseline, posttreatment	BBT PPT ROM MAS 2PD NSA SIS FMA-UE	Significant differences in ROM shoulder ABD and elbow EXT (*p* = 0.04) Improvement of BBT (*p* = 0.03), FM-UE (*p* = 0.03), speed and motor coordination (*p* = 0.05)

[25]	Design: RCT To investigate whether MI training has a positive influence on upper extremity performance in stroke patients	Stage: chronic *n* = 24 *n* (IG) = 12 *n* (CG) = 12	4 wk IG: 30min × 3t/wk MI + 30min × 5t/wk FT CG: 30min × 3t/wk MI + 30min × 5t/wk FT Assessment: baseline, posttreatment	FMA-UE WMFT	FMA-UE: improve 8.17 pt in IG WMFT: improve 6.25 pt in IG

[26]	Design: RCT Evaluated motor function of the upper extremity and investigated neural plastic changes before and after treatment using diffusion tensor imaging and transcranial magnetic stimulation	Stage: subacute *n*: 20 *n* (IG): 10 *n* (CG): 10	5t/wk × 4wk IG: 45 min MIT + 45min traditional rehabilitation CG: 45 min traditional rehabilitation Assessment: baseline, posttreatment	FMA-UE ARAT TMS	Better score in ARAT for IG (6.48) Significant improvement in FMA-UE for IG (4.7)

[27]	Design: RCT To evaluate whether combining MP with physical practice training enhances hand function in patients with stroke	Stage: subacute *n*: 20 *n* (IG): 10 *n* (CG): 10	5 d/wk × 4 wks IG: 45 min Bobath + 45 min × 3 ss with 5 min rest between 2 ss PM-IM CG: 45 min Bobath Assessment: baseline, posttreatment	ARAT fMRI Activated voxels of SMC	Significant difference in both groups for ARAT (*p* = 0.042) Significant improvement between pre- and posttreatment (*p* = 0.001) Increase in ARAT of 12.65 for IG and 5.20 for CG

[28]	Design: RCT To investigate the adjuvant effects of MP using an inverse video of the unaffected limb in subacute stroke patients with severe motor impairment on motor improvement, functional outcomes, and activities of daily living	Stage: subacute *n* = 20 *n* (IG) = 10 *n* (CG) = 10	5t/wk × 4wk IG: 30 min rehabilitation + 20min MP inverse video of the unaffected limb CG: 30 min rehabilitation Assessment: baseline, 4 wk	FMA-UE MFT FIM	No significant differences in all outcomes between groups Significant differences in FMA-UE and FIM posttreatment in both groups

[29]	Design: RCT To determine whether the imagery perspective used during MP differentially influenced performance outcomes after stroke	Stage: chronic *n* = 19 *n* (IGint) = 6 *n* (IGext) = 7 *n* (CG) = 6	2t/wk × 6wk IGint: 30 min occupational therapy + MP internal perception IGext: 30 min occupational therapy + MP external perception CG: 30 min occupational therapy + relaxation imagery training Assessment: baseline and posttreatment	FMA-UE JTTHF COPM	Significant improvement in IGint and IGext Significant improvement in all the groups for COPM (*p* < 0.05) Improvement in FMA for all groups, but only significant for IGint (*M* 5 9.6, SEM 5 1.03) and IGext (*M* 5 10.6, SEM 5 2.94) For self-perception of performance, COPM mean improve (*p* < 0.001): CG 12.3 (SEM 5 3.86), IGint 13.2 (SEM 5 3.09), IGext 15.6 (SEM 5 3.79)

[30]	Design: RCT To investigate the effects of adjuvant MP on affected upper limb function following a stroke using three-dimensional (3D) motion analysis	Stage: subacute *n* = 10 *n* (IGa) = 5 *n* (IGb) = 5	IGa: 3wk of MP + conventional rehabilitation therapy; 3 wk conventional rehabilitation therapy IGb: 3 wk conventional rehabilitation therapy; 3 wk of MP + conventional rehabilitation therapy MP: 20min × 3t/wk Assessment: baseline, posttreatment, 3 wk, 6 wk	3D motion analysis FMA-UE MAL-30	No significant differences between groups during assessment of effect and treatment period No significant differences in comparisons between groups analyzing 3D movement and comparisons between groups on rating scales

[31]	Design: RCT Compared efficacy of a “massed” MP regimen versus a “distributed” MP regimen on upper extremity motor impairment and functional limitation	Stage: chronic *n*: 27 *n* IGm: 13 *n* IGd: 14	3 t/wk × 10 wk 60min PM + 1/2 TC IGm: 30 min exercise + 5 min Jacobson relaxation + 60min MP in audio IGd: 30 min exercise + 5 min Jacobson relaxation + 20min of MP in audio + 2 more phases at home Assessment: baseline, 10 wk and 3 m	FMA-UE ARAT	IGd more significant improvement than IGm (*p* < 0.001) at 10 wk Significant difference in ARAT at 3 m for IGd

[32]	Design: RCT To investigate the role of MP in functional recovery of upper limbs in stroke patients	Stage: subacute *n* = 36 *n* (IGa) = 18 *n* (IGb) = 18	IGa: 3h/d × 5d × 3wk of conventional neurorehabilitation protocol (therapeutic exercise and occupational therapy) + 60min of MP IGb: 3wk of rehabilitation program + MP + 3k conventional neurorehabilitation protocol Assessment: baseline, posttreatment, 3 wk, 6 wk	MI AFT	No significant differences posttreatment Significant differences between groups at 3 wks Difference was minimal at 6 wks

[33]	Design: RCT To evaluate the effectiveness of a task-oriented MP approach as an addition to regular arm-hand therapy in patients with subacute stroke	Stage: subacute *n* = 42 *n* (IG) = 21 *n* (CG) = 21	Training: 10 min × 3t/d × 6wk IG: conventional therapy + MP instruction video CG: Bobath + exercise program Assessment: baseline, posttreatment, 3 follow-ups for 1 year and 12 months	FMA-UE FAT WMFT Accelerometry	Improvement on FMA-UE and WMFT in both groups Significant improvement on FAT test posttreatment and maintain during 12 months on IG No significant differences between groups on training effect

[34]	Design: RCT To identify the targets for MI in stroke rehabilitation from a voxel-based whole brain analysis of resting-state functional magnetic resonance imaging	Stage: chronic *n* = 34 *n* (IG): 17 *n* (CG): 17	3h/d × 5d/wk × 4wk IG: 30 min MIT + conventional rehabilitation CG: 30 min stroke education conventional rehabilitation Assessment: baseline, posttreatment	FMA-UE mBI MRI	Significant improvement for IG in FMA-UE (CG: 21.1 ± 16.4, IG: 33.3 ± 14.3, *p* = 0.02) Positive correlation between slow-5 band in the ipsilesional IPL and FM-UE Different alternative for functional connectivity in IG for ipsilesional IPL that correlated positively with FM-UL MI rehabilitation efficiency was associated with an increased slow-5 band and impaired functional connectivity in ipsilesional IPL

2PT: 2-Point Test; ADL: activities of daily living; AFT: Arm Functional Test; ARAT: Action Research Arm Test; AO: Action-Observation; BBT: Box and Blocks Test; CG: control group; COPM: Canadian Occupational Performance Measure; d: days; CT: clinical trial; FAT: Frenchay Arm Test; FMA-UE: Fugl-Meyer Assessment Upper Extremity; FIM: Functional Independence Measure; fMRI: functional magnetic resonance imaging; MRI: magnetic resonance imaging; IG: Intervention Group; JTHFT: Jebsen and Taylor Hand Function Test; MAL: Motor Activity Log; MAL AOU: Motor Activity Log Amount of Use; MAL QOM: Motor Activity Log Quality of Movement; m: month; MAS: Modified Ashworth Scale; mBI: modified Barthel Index; MCID: Minimal Clinically Important Difference; MFT: Motor Function Test; MI: motor imagery; min: minutes; MP: mental practice; *n*: number; NSA: Nottingham Sensory Assessment; PG: Placebo Group; PPT: Purde-Pegboard Test; pt: points; RCT: randomized clinical trial; ROM: Range Of Movement; SIS: Stroke Impact Scale; ss: sessions; *t*: time; TMS: Transcraneal Magnetic Stimulation; WMFT: Wolf Motor Function Test; wk: weeks.

The article "Motor Imagery and Mental Practice in the Subacute and Chronic Phases in Upper Limb Rehabilitation after Stroke: A Systematic Review" was published in 2023. Journal: Occup Ther Int.

**Table 2:** Assessment of the methodological quality of the studies using the PEDRo scale.

	Randomization	Hidden assignment	Groups homogeneous	Subjects blinded	Therapists blinded	Evaluators blinded	Follow-up subjects	Intention to treat	Comparison between groups	Scoring and variability measures	Total
[37]	0	0	1	0	0	0	1	1	1	1	5
[47]	1	0	1	0	0	0	1	1	1	1	6
[41]	1	0	1	0	0	1	1	1	1	1	7
[42]	1	1	1	0	0	1	1	0	1	1	7
[45]	1	0	1	0	0	1	1	0	1	1	6
[40]	1	1	1	0	0	0	0	1	1	1	6
[43]	1	1	0	1	0	1	1	1	1	1	8
[38]	1	1	1	0	0	1	0	0	1	1	6
[46]	1	1	0	0	0	0	1	1	1	1	6
[39]	1	1	1	0	0	1	1	0	1	1	7
[44]	1	1	1	0	1	0	1	0	1	1	7

## Data Availability

The data of the study are available from the corresponding author.

## References

[1] OMS (2017). https://www.who.int/es/news-room/fact-sheets/detail/cardiovascular-diseases-(cvds).

[2] Moyano Á. (2010). El accidente cerebrovascular desde la mirada del rehabilitador. *Revista Hospital Clínica Universidad de Chile*.

[3] Ruiz-Ares G., Martínez-Sánchez P., Fuentes B. (2015). Cerebrovascular diseases. *Medicine*.

[4] Bernhardt J., Hayward K. S., Kwakkel G. (2017). Agreed definitions and a shared vision for new standards in stroke recovery research: the Stroke Recovery and Rehabilitation Roundtable taskforce. *Neurorehabilitation and Neural Repair*.

[5] Fernández Gómez E., Sánchez Cabeza Á. (2018). Imaginería motora: revisión sistemática de su efectividad en la rehabilitación de la extremidad superior tras un ictus. *Revista de Neurologia*.

[6] Kwon J.-S., Park M.-J., Yoon I.-J., Park S.-H. (2012). Effects of virtual reality on upper extremity function and activities of daily living performance in acute stroke: a double-blind randomized clinical trial. *Neuro Rehabilitation*.

[7] Copper C., Moran A., Driskell J. E. (1994). Does mental practice enhance performance?. *Journal of Applied Psychology*.

[8] Decety J. (1996). The neurophysiological basis of motor imagery. *Behavioural Brain Research*.

[9] Jeannerod M. (1994). The representing brain: neural correlates of motor intention and imagery. *Behavioral and Brain Sciences*.

[10] Malouin F., Belleville S., Richards C. L., Desrosiers J., Doyon J. (2004). Working memory and mental practice outcomes after stroke^1^. *Archives of Physical Medicine and Rehabilitation*.

[11] Deiber M. P., Ibañez V., Honda M., Sadato N., Raman R., Hallett M. (1998). Cerebral processes related to visuomotor imagery and generation of simple finger movements studied with positron emission tomography. *Neuro Image*.

[12] Gowda A. S., Memon A. N., Bidika E., Salib M., Rallabhandi B., Fayyaz H. (2021). Investigating the viability of motor imagery as a physical rehabilitation treatment for patients with stroke-induced motor cortical damage. *Cureus*.

[13] Errante A., Bozzetti F., Sghedoni S. (2019). Explicit motor imagery for grasping actions in children with spastic unilateral cerebral palsy. *Frontiers in Neurology*.

[14] Borges L. R., Fernandes A. B., Melo L. P., Guerra R. O., Campos T. F. (2018). Action observation for upper limb rehabilitation after stroke. *Cochrane Database of Systematic Reviews*.

[15] Yágüez L., Nagel D., Hoffman H., Canavan A. G. M., Wist E., Hömberg V. (1998). A mental route to motor learning: improving trajectorial kinematics through imagery training. *Behavioural Brain Research*.

The article "Motor Imagery and Mental Practice in the Subacute and Chronic Phases in Upper Limb Rehabilitation after Stroke: A Systematic Review" was published in 2023. Journal: Occup Ther Int.

[16] Nilsen D. M., Gillen G., Gordon A. M. (2010). Use of mental practice to improve upper-limb recovery after stroke: a systematic review. *American Journal of Occupational Therapy*.

[17] Kosslyn S. M., Cacioppo J. T., Davidson R. J. (2002). Bridging psychology and biology: the analysis of individuals in groups. *American Psychologist*.

[18] Bai O., Huang D., Fei D. Y., Kunz R. (2014). Effect of real-time cortical feedback in motor imagery-based mental practice training. *Neuro Rehabilitation*.

[19] Kraft E., Schaal M. C., Lule D., Koenig E., Scheidtmann K. (2015). The functional anatomy of motor imagery after sub-acute stroke. *NeuroRehabilitation*.

[20] Wang H., Xu G., Wang X. (2019). The reorganization of resting-state brain networks associated with motor imagery training in chronic stroke patients. *IEEE Transactions on Neural Systems and Rehabilitation Engineering*.

[21] Smith V., Devane D., Begley C. M., Clarke M. (2011). Methodology in conducting a systematic review of systematic reviews of healthcare interventions. *BMC Medical Research Methodology*.

[22] Page M. J., McKenzie J. E., Bossuyt P. M. (2021). The PRISMA 2020 statement: an updated guideline for reporting systematic reviews. *BMJ*.

[23] Timmermans A. A. A., Verbunt J. A., van Woerden R., Moennekens M., Pernot D. H., Seelen H. A. M. (2013). Effect of mental practice on the improvement of function and daily activity performance of the upper extremity in patients with subacute stroke: a randomized clinical trial. *Journal of the American Medical Directors Association*.

[24] Oh H. S., Kim E. J., Kim D. Y., Kim S. J. (2016). Effects of adjuvant mental practice on affected upper limb function following a stroke: results of three-dimensional motion analysis, Fugl-Meyer assessment of the upper extremity and motor activity logs. *Annals of Rehabilitation Medicine*.

[25] Riccio I., Iolascon G., Barillari M. R., Gimigliano R., Gimigliano F. (2010). Mental practice is effective in upper limb recovery after stroke: a randomized single-blind cross-over study. *European Journal of Physical and Rehabilitation Medicine*.

[26] Liu H., Song L. P., Zhang T. (2014). Mental practice combined with physical practice to enhance hand recovery in stroke patients. *Behavioural Neurology*.

[27] Nam J. S., Yi T. I., Moon H. I. (2019). Effects of adjuvant mental practice using inverse video of the unaffected upper limb in subacute stroke: a pilot randomized controlled study. *International Journal of Rehabilitation Research. Internationale Zeitschrift Fur Rehabilitationsforschung. Revue Internationale de Recherches de Readaptation*.

The article "Motor Imagery and Mental Practice in the Subacute and Chronic Phases in Upper Limb Rehabilitation after Stroke: A Systematic Review" was published in 2023. Journal: Occup Ther Int.

[28] Nilsen D. M., Gillen G., DiRusso T., Gordon A. M. (2012). Effect of imagery perspective on occupational performance after stroke: a randomized controlled trial. *The American Journal of Occupational Therapy*.

[29] Kim S.-S., Lee B.-H. (2015). Motor imagery training improves upper extremity performance in stroke patients. *Journal of Physical Therapy Science*.

[30] Page S. J., Hade E. M., Pang J., Sciences R., Ohio T. (2017). Retention of the spacing effect with mental practice in hemiparetic stroke. *Experimental Brain Research*.

[31] Azad A., Mahmoodi-Manbar A., Arani-Kashani Z. (2018). Effect of motor imagery training with sensory feedback on sensory-motor function of the upper extremity in patients with chronic stroke. *Journal of Babol University of Medical Sciences*.

[32] Wang X., Wang H., Xiong X. (2020). Motor imagery training after stroke increases Slow-5 oscillations and functional connectivity in the Ipsilesional inferior parietal lobule. *Neurorehabilitation and Neural Repair*.

[33] de Morton N. A. (2009). The PEDro scale is a valid measure of the methodological quality of clinical trials: a demographic study. *The Australian Journal of Physiotherapy*.

[34] Maher C. G., Sherrington C., Herbert R. D., Moseley A. M., Elkins M. (2003). Reliability of the PEDro scale for rating quality of randomized controlled trials. *Physical Therapy*.

[35] Li F., Zhang T., Li B.-J., Zhang W., Zhao J., Song L.-P. (2018). Motor imagery training induces changes in brain neural networks in stroke patients. *Neural Regeneration Research*.

[36] Kim H., Yoo E. Y., Jung M. Y., Kim J., Park J. H., Kang D. H. (2018). The effects of mental practice combined with modified constraint-induced therapy on corticospinal excitability, movement quality, function, and activities of daily living in persons with stroke. *Disability and Rehabilitation*.

[37] Krakauer J. W. (2005). Arm function after stroke: from physiology to recovery. *Seminars in Neurology*.

[38] Thieme H., Bayn M., Wurg M., Zange C., Pohl M., Behrens J. (2013). Mirror therapy for patients with severe arm paresis after stroke – a randomized controlled trial. *Clinical Rehabilitation*.

[39] Machado S., Lattari E., de Sa A. (2015). Is mental practice an effective adjunct therapeutic strategy for upper limb motor restoration after stroke? A systematic review and meta- analysis. *CNS & Neurological Disorders-Drug Targets*.

[40] Monte-Silva K. (2013). Effects of tDCS combined with mcimt or mental practice in poststroke patients. https://Clinicaltrials.Gov/Show/Nct01879787.

[41] Monteiro K. B., dos Santos Cardoso M., da Costa Cabral V. R. (2021). Effects of motor imagery as a complementary resource on the rehabilitation of stroke patients: a meta-analysis of randomized trials. *Journal of Stroke and Cerebrovascular Diseases*.

The article "Motor Imagery and Mental Practice in the Subacute and Chronic Phases in Upper Limb Rehabilitation after Stroke: A Systematic Review" was published in 2023. Journal: Occup Ther Int.

[42] Stockley R. C., Jarvis K., Boland P., Clegg A. J. (2021). Systematic review and meta-analysis of the effectiveness of mental practice for the upper limb after stroke: Imagined or real benefit?. *Archives of Physical Medicine and Rehabilitation*.

[43] Barclay R. E., Stevenson T. J., Poluha W., Semenko B., Schubert J. (2020). Mental practice for treating upper extremity deficits in individuals with hemiparesis after stroke. *Cochrane Database of Systematic Reviews*.

[44] Melogno M., Nunez S., Landa S. (2017). Revisión sistemática sobre instrumentos de valoración de la imaginación motora para población hispanohablante: su uso en rehabilitación. *Revista de Neurologia*.

[45] Stinear C. M., Byblow W. D., Steyvers M., Levin O., Swinnen S. P. (2006). Kinesthetic, but not visual, motor imagery modulates corticomotor excitability. *Experimental Brain Research*.

[46] Johnson S. H., Sprehn G., Saykin A. J. (2002). Intact motor imagery in chronic upper limb hemiplegics: evidence for activity-independent action representations. *Journal of Cognitive Neuroscience*.

[47] Sirigu A., Duhamel J. R., Cohen L., Pillon B., Dubois B., Agid Y. (1996). The mental representation of hand movements after parietal cortex damage. *Science*.

[48] Sirigu A., Duhamel J. R. (2001). Motor and visual imagery as two complementary but neurally dissociable mental processes. *Journal of Cognitive Neuroscience*.

[49] Bovend’Eerdt T. J., Dawes H., Sackley C., Izadi H., Wade D. T. (2010). An integrated motor imagery program to improve functional task performance in neurorehabilitation: a single-blind randomized controlled trial. *Archives of Physical Medicine and Rehabilitation*.

